# The Influence of Mixed Teaching Mode on the Learning Effects of Psychology Students' Experiment Course in Higher Vocational Colleges

**DOI:** 10.1155/2022/4190668

**Published:** 2022-03-08

**Authors:** Haiying Quan, Zimeng Guo, Rongjing Ni, Chen Li, Xin Deng

**Affiliations:** ^1^School of Physical Education, Liaoning Normal University, Liaoning, Dalian 116029, China; ^2^Department of Physical Education, Harbin Engineering University, Heilongjiang, Haerbin 150001, China

## Abstract

In this paper, we are going to analyze the influence of mixed teaching mode on the teaching effect of psychology students' experiment courses in higher vocational colleges. To realize and verify these claims, 80 psychology students of grade 2020 in our school were selected for observation. Class 1 of the psychology major in our school was randomly selected as the observation group (*n* = 40) and Class 2 as the control group (*n* = 40). The mixed teaching mode and the traditional teaching mode were adopted, respectively. After intervention, the experimental examination results, experimental report score, general evaluation results of the experiment, and experimental pass rate of the observation group were higher than those before intervention (*P* < 0.05). The control group had no significant change before and after intervention (*P* > 0.05). The experimental examination results, experimental report score, general evaluation results of the experiment, and experimental pass rate of the observation group were all higher than those of the control group, with statistical significance (*P* < 0.05). The results show that in the observation group, 92.50% of the students believed that the mixed teaching mode could arouse the enthusiasm for learning and improve the activity of the experimental class. 97.50% of the students thought that the mixed teaching mode could stimulate students' interest in learning and improve the ability of experimental operation. 100.00% of the students thought the mixed teaching mode could be helpful in understanding the experimental. The evaluation result of the teaching mode was significantly higher than that of the control group, and the comparison result was statistically significant (*P* < 0.05). After receiving the mixed teaching mode, the observation group had a higher satisfaction with the teaching effect, with a satisfaction rate of 95.00%. The control group had low satisfaction with the teaching effect, with a satisfaction rate of 52.50%, and the difference was statistically significant (*P* < 0.05). Through the application of the mixed teaching mode combining online and offline, psychology students in higher vocational colleges can achieve better learning results and improve students' evaluation and satisfaction of teaching effect of the mixed teaching mode of psychology experiment teaching mode in higher vocational colleges.

## 1. Introduction

The teaching courses of psychology major in higher vocational colleges can be roughly divided into two kinds, namely, theory type and practice type [1]. For theoretical psychology courses, the traditional teaching style supplemented by an assisted teaching mode can meet the cognitive needs of students for many theories [2, 3]. As for practical psychology courses, they are only limited to the teacher's explanation of the theory in class, so students cannot learn the theory to the maximum extent and cannot use the theory well to solve problems in reality [4]. The experiment course is the main representative of practical psychology courses in higher vocational colleges. Therefore, the traditional teaching mode has been unable to guarantee the teaching effect, and it is necessary to apply the teaching mode in line with the needs of the times and meet the needs of the experimental teaching effect of psychology students in higher vocational colleges [5, 6]. In recent years, the rapid development of information technology has promoted the continuous reform and improvement of the teaching mode of psychology students' experiment courses in higher vocational colleges. Mixed teaching should always adhere to the concept of student-centered, goal-oriented, and continuous improvement [7]. In the course of teaching design, online and offline teaching modes should be combined [8]. Mixed teaching combines the essence of various psychological theories, such as humanistic learning theory, that is, teachers should pay attention not only to the cognitive development of students in the teaching process but also to the exploration of students' inner worlds, so as to achieve the purpose of matching the application of methods in the teaching process with students' hobbies, needs, experiences and personality differences. Finally, it can not only stimulate students' cognitive and behavioral potential but also promote their creativity level [9, 10]. In order to explore the influence of mixed teaching modes on the teaching effect of an experimental course for psychology students in higher vocational colleges, 80 psychology students of grade 2020 in our school were selected for observation in this study.

In this paper, we are going to analyze the influence of mixed teaching mode on the teaching effect of psychology students' experiment courses in higher vocational colleges. To realize and verify these claims, 80 psychology students of grade 2020 in our school were selected for observation. Class 1 of the psychology major in our school was randomly selected as the observation group (*n* = 40) and Class 2 as the control group (*n* = 40). The mixed teaching mode and the traditional teaching mode were adopted, respectively. After intervention, the experimental examination results, experimental report score, general evaluation results of the experiment, and experimental pass rate of the observation group were higher than those before intervention (*P* < 0.05). The control group had no significant change before and after intervention (*P* > 0.05). The experimental examination results, experimental report score, general evaluation results of the experiment, and experimental pass rate of the observation group were all higher than those of the control group, with statistical significance (*P* < 0.05).

The rest of the manuscript is arranged as follows: In the subsequent section, the proposed methodology, which is used to measure the effects of the teaching, is presented along with sufficient detailed information about its structure, organization, and implementation plan. Experimental results and observations of the proposed approach in the real environment of colleges are presented both in textual and graphical formats whenever applicable and possible. In addition, a generalized discussion section is provided to provide all this information in a summarized form. Lastly, concluding remarks are given.

## 2. Proposed Method or Approach

### 2.1. General Information

80 psychology students of grade 2020 in our school were selected for observation. Class 1 of the psychology major in our school was randomly selected as the observation group (*n* = 40) and Class 2 as the control group (*n* = 40). The mixed teaching mode and the traditional teaching mode were adopted, respectively. The experimental instruments, teaching hours, teaching syllabus, and experimental courses of the observation group and the control group were consistent. There was no significant difference between the two groups in age, gender, and scores of the last experiment (*P* > 0.05).

Inclusion criteria were as follows:

1. Students majoring in psychology in our school
2. Those not divorced from the research during the research period
3. Those who voluntarily participated in the study and signed the informed consent

Exclusion criteria were as follows:

1. Those who actively applied for withdrawal from the study
2. Those who voluntarily applied to withdraw from this research

There was no significant difference in general data between the two groups (*P* > 0.05), indicating comparability. With the approval of the Ethics Committee of our school, the general information of the two groups is as shown in Table 1.

### 2.2. Methodology

The control group was given a traditional teaching mode, including routine preparation before class and using PPT to explain the experimental content, and then, the teacher taught the experimental operation. After class, the students reviewed the contents of the experimental lesson according to the requirements of the teacher.

The observation group was given a mixed teaching mode, including online learning and offline learning. Teachers chose appropriate online learning resources according to the requirements in the syllabus and course standards and students' conditions and then conducted experimental teaching after processing or self-making:

1. Before class: released preview courseware, inserted voice prompts for important and difficult points; pushed relevant network learning resources. By checking the background data, teachers urged the students who had not completed the preview, grasped the situation of students' preview, and planned the focus of classroom teaching in advance.
2. During class: students scanned the randomly generated QR code to check in to class. Teachers shared courseware to students' mobile phones. During the experimental operation, students could repeatedly check the experimental operation demonstration video inserted in the courseware. The interaction between teachers and students would be carried out through a variety of forms, such as time-limited quizzes, online answering, and random roll calls [11].
3. After class: through analysis and feedback of learning data, teachers could understand students' learning situations point-to-point and answer questions online and offline in a timely manner in response to questions raised by students. According to the experimental results, students completed the experimental report, and teachers assessed students' grades based on their online and offline performance.

### 2.3. Observational Index

The intervention time of the two groups was 1month, and the observation indexes of the two groups were compared, including the following:

1. Learning effect: experimental examination results, experimental report score, general evaluation results of the experiment, and experimental pass rate.
2. Evaluation of teaching model effect: arousing the enthusiasm for learning, improving the activity of experimental class, stimulating students' interest in learning, being helpful in understanding the experimental knowledge, and improving the ability of experimental operation [12]. The evaluation level was divided into four parts: strongly agree, agree, disagree, and strongly disagree. The calculation formula of agreement was agreement = strongly agree + agree/total number of cases.
3. Teaching affect satisfaction: the evaluation was conducted at three levels: very satisfied, relatively satisfied, and dissatisfied. The satisfaction calculation formula was satisfaction = very satisfied + relatively satisfied/total number of cases.

### 2.4. Statistical Method

The results of this study were analyzed and processed by SPSS25.0 software, and the measurement data were expressed as mean ± standard deviation. The independent sample *t*-test was used for comparison between groups, and enumeration data were expressed as frequency and rate (*n*(%)). *P* < 0.05 indicated that the data difference is statistically significant.

## 3. Experimental Results and Observations

### 3.1. Contrast Results of Learning Effect

After intervention, the experimental examination results, experimental report score, general evaluation results of the experiment, and experimental pass rate of the observation group were higher than those before intervention (*P* < 0.05). The control group had no significant change before and after intervention (*P* > 0.05). The experimental examination results, experimental report score, general evaluation results of the experiment, and experimental pass rate of the observation group were all higher than those of the control group, with statistical significance (*P* < 0.05). Contrast results of the learning effect are shown in Table 2.

### 3.2. Contrast Results of Evaluation of Teaching Modal Effect

The results show that in the observation group, 92.50% of the students believed that the mixed teaching mode could arouse the enthusiasm for learning and improve the activity of the experimental class. 97.50% of the students thought that the mixed teaching mode could stimulate students' interest in learning and improve the ability of experimental operation. 100.00% of the students thought the mixed teaching mode could be helpful in understanding the experimental. The evaluation result of the teaching mode was significantly higher than that of the control group, and the comparison result was statistically significant (*P* < 0.05). Contrast results of the evaluation of the teaching modal effect are shown in Table 3.

### 3.3. Contrast Results of Evaluation of Teaching Effect Satisfaction

After receiving the mixed teaching mode, the observation group had a higher satisfaction with the teaching effect, with a satisfaction rate of 95.00%. The control group had low satisfaction with the teaching effect, with a satisfaction rate of 52.50%, and the difference was statistically significant (*P* < 0.05). Contrast results of the evaluation of teaching effect satisfaction are shown in Table 4.

## 4. Discussion

With the great development of social economy in China, the daily life of psychology students in higher vocational colleges has become increasingly rich and contact with high-tech things has become a routine [13, 14]. Compared with the colorful life of psychology students in higher vocational colleges, if college teachers still use the traditional teaching mode of “teachers speak all the words” to teach psychology students, it is bound to reduce their interest in the course [15]. Therefore, under the background of “Internet +” education, the reform of the traditional teaching mode is imperative [16]. The mixed teaching mode combines the advantages of traditional teaching and online learning, which not only give full play to the leading role of teachers in guiding, inspiring, and monitoring the teaching process but also fully reflect the initiative, enthusiasm, and creativity of students as the main body of the learning process [17, 18]. Mixed teaching will become the new normal in the postepidemic era. It requires the participation of schools, teachers, and students. The comprehensive deployment of mixed teaching at the school level, the formulation of relevant policies, and the strengthening of training can promote the extensive implementation of the mixed teaching mode [19]. As the main implementer of blended teaching, teachers should pay attention to guiding students, using a variety of teaching methods, stimulating students' learning enthusiasm, so as to achieve the ultimate goal of improving students' learning experience and enhancing students' learning effect [20, 21].

The results of this study showed that after intervention, the experimental examination results, experimental report score, general evaluation results of the experiment, and experimental pass rate of the observation group were higher than those before intervention (*P* < 0.05). The control group has no significant change before and after intervention (*P* > 0.05). The experimental examination results, experimental report score, general evaluation results of the experiment, and experimental pass rate of the observation group were all higher than those of the control group, with statistical significance (*P* < 0.05). The results show that in the observation group, 92.50% of the students believed that the mixed teaching mode could arouse the enthusiasm for learning and improve the activity of the experimental class. 97.50% of the students thought that the mixed teaching mode could stimulate students' interest in learning and improve the ability of experimental operation. 100.00% of the students thought the mixed teaching mode could be helpful in understanding the experimental. The evaluation result of the teaching mode was significantly higher than that of the control group, and the comparison result was statistically significant (*P* < 0.05). After receiving the mixed teaching mode, the observation group had higher satisfaction with the teaching effect, with a satisfaction rate of 95.00%. The control group had low satisfaction with the teaching effect, with a satisfaction rate of 52.50%, and the difference was statistically significant (*P* < 0.05).

## 5. Conclusion

In this paper, we analyzed the influence of mixed teaching mode on the teaching effect of psychology students' experiment courses in higher vocational colleges. To realize and verify these claims, 80 psychology students of grade 2020 in our school were selected for observation. Class 1 of the psychology major in our school was randomly selected as the observation group (*n* = 40) and Class 2 as the control group (*n* = 40). The mixed teaching mode and the traditional teaching mode were adopted, respectively. After intervention, the experimental examination results, experimental report score, general evaluation results of the experiment, and experimental pass rate of the observation group were higher than those before intervention (*P* < 0.05). The control group had no significant change before and after intervention (*P* > 0.05). The experimental examination results, experimental report score, general evaluation results of the experiment, and experimental pass rate of the observation group were all higher than those of the control group, with statistical significance (*P* < 0.05). Finally, through the application of the mixed teaching mode combining online and offline, psychology students in higher vocational colleges can achieve better learning results and improve their evaluation and satisfaction of teaching effect of the mixed teaching mode of psychology experiment teaching mode in higher vocational colleges.

## Figures and Tables

**Table 1:** General information of two groups.

General information		Observation group	Control group	*P*
Cases		40	40	>0.05
Gender	Male	16	19	>0.05
	Female	24	21	
Age (average)		19.25 ± 1.09	19.17 ± 1.25	>0.05
Scores of the last experiment	Experimental examination results	67.82 ± 3.07	66.89 ± 4.12	>0.05
	Experimental report score	63.45 ± 5.96	64.21 ± 6.17	
	General evaluation results of the experiment	66.32 ± 5.22	65.97 ± 5.49	
	Experimental pass rate	11 (27.50%)	12 (30.00%)	

**Table 2:** Contrast results of learning effect.

Groups		Observation group	Control group	t	*P*
Experimental examination results	Before intervention	67.82 ± 3.07	66.89 ± 4.12	0.328	>0.05
	After intervention	91.05 ± 2.62	70.24 ± 6.28	7.569	<0.05
Experimental report score	Before intervention	63.45 ± 5.96	64.21 ± 6.17	0.526	>0.05
	After intervention	84.81 ± 8.46	65.27 ± 4.51	5.267	<0.05
General evaluation results of the experiment	Before intervention	66.32 ± 5.22	65.97 ± 5.49	0.248	>0.05
	After intervention	89.70 ± 2.45	64.38 ± 5.21	9.541	<0.05
Experimental pass rate	Before intervention	11 (27.50%)	12 (30.00%)	0.336	>0.05
	After intervention	34 (85.00)	16 (40.00)	8.156	<0.05

**Table 3:** Contrast results of evaluation of teaching modal effect.

Groups		Strongly agree	Agree	Disagree	Strongly disagree	Agreement (%)	*P*
Arousing the enthusiasm for learning	Observation group	14	23	3	0	92.50	<0.05
	Control group	9	11	8	12	50.00	
Improving the activity of the experimental class	Observation group	12	25	2	1	92.50	<0.05
	Control group	7	14	11	8	52.50	
Stimulating students' interest in learning	Observation group	15	24	1	0	97.50	<0.05
	Control group	9	12	10	9	52.50	
Being helpful in understanding the experimental knowledge	Observation group	19	21	0	0	100.00	<0.05
	Control group	10	12	10	8	55.00	
Improving the ability of experimental operation	Observation group	14	25	0	1	97.50	<0.05
	Control group	8	10	12	10	45.00	

**Table 4:** Contrast results of evaluation of teaching effect satisfaction.

Groups		Very satisfied	Relatively satisfied	Dissatisfied	Satisfaction (%)
Observation group	40	14	24	2	95.00
Control group	40	8	13	19	52.50
*P*		<0.05	<0.05	<0.05	<0.05

## Data Availability

The data used to support the findings of this study are included within the article.
